RETRACTED

# Enhancing radiosensitivity of melanoma cells through very high dose rate pulses released by a plasma focus device

**DOI:** 10.1371/journal.pone.0199312

**Published:** 2018-06-29

**Authors:** Francesca Buontempo, Ester Orsini, Isabella Zironi, Lorenzo Isolan, Alessandra Cappellini, Stefania Rapino, Agostino Tartari, Domiziano Mostacci, Giorgio Cucchi, Alberto Maria Martelli, Marco Sumini, Gastone Castellani

**Affiliations:** 1 University of Bologna, Department of Biomedical and Neuromotor Sciences, Bologna, Italy; 2 University of Bologna, Department of Physics and Astronomy, Bologna, Italy; 3 University of Bologna, Department of Chemistry “G. Ciamician”, Bologna, Italy; 4 Interdepartmental Centre “L. Galvani” (CIG) for integrated studies of bioinformatics, biophysics and biocomplexity, Bologna, Italy; 5 European Institute of Oncology and Monzino Cardiac Center Foundation (IEO-CCM), Milano, Italy; 6 University of Bologna, Department of Industrial Engineering, Bologna, Italy; 7 University of Cassino and Southern Lazio, Department of Human Social and Health Sciences, Cassino, Italy; 8 National Institute for Nuclear Physics (INFN), Bologna, Italy; Northwestern University Feinberg School of Medicine, UNITED STATES

## Abstract

Radiation therapy is a useful and standard tumor treatment strategy. Despite recent advances in delivery of ionizing radiation, survival rates for some cancer patients are still low because of recurrence and radioresistance. This is why many novel approaches have been explored to improve radiotherapy outcome. Some strategies are focused on enhancement of accuracy in ionizing radiation delivery and on the generation of greater radiation beams, for example with a higher dose rate. In the present study we proposed an *in vitro* research of the biological effects of very high dose rate beam on SK-Mel28 and A375, two radioresistant human melanoma cell lines. The beam was delivered by a pulsed plasma device, a “Mather type” Plasma Focus for medical applications. We hypothesized that this pulsed X-rays generator is significantly more effective to impair melanoma cells survival compared to conventional X-ray tube. Very high dose rate treatments were able to reduce clonogenic efficiency of SK-Mel28 and A375 more than the X-ray tube and to induce a greater, less easy-to-repair DNA double-strand breaks. Very little is known about biological consequences of such dose rate. Our characterization is preliminary but is the first step toward future clinical considerations.

## Introduction

Radiation therapy (RT) is a key component of cancer treatment; approximately 50% of all patients with cancer receive RT at some points during the course of treatment, alone or in combination with surgery and/or chemotherapy [1–3]. Although this local treatment modality may improve survival and quality of patients’ life even in late stages of their disease, a large fraction of them subsequently develops radioresistance and recurrence [1, 4, 5]. Novel strategies are urgently needed to overcome tumor radioresistance and thus improve RT outcome. In the last decade, many studies have been aimed at enhancing biological effects of radiotherapy according to two main approaches. One, biologic, is related to radiosensitization of tumor cells (without sensitizing normal tissue cells), mostly through targeted and immune therapies [6–11]. The other one, technologic, is more focused on improvement of accuracy in delivering ionizing radiation (IR) and on generation of greater radiation beams, for example with a higher dose rate (DR), to counteract radioresistance [3, 12–18]. DR, the quantity of radiation absorbed per unit time, is one of the principal factors determining the biological consequences of a given absorbed dose. As the DR is increased and the exposure time reduced, the biological effects are generally more significant [12, 19, 20]. A number of *in vitro* studies have been conducted and a wide range of DRs has been used, between the seventies and the nineties, to assess the low-Linear Energy Transfer (LET) dose-rate effect. In general, it was observed that the cell killing effect of X or γ rays decreased continuously as the dose-rate decreased due to repair of sub-lethal damage taking place during irradiation [21]. At lower dose-rates, cell proliferation continued during irradiation and the ultimate outcome was a complex overlapping of cellular radiosensitivity, dose/cell cycle and tissue adaptability [19, 22, 23]. However, concerning the very high dose-rates, the state of knowledge of mammalian cells exposition was not so evident [20]. Recent developments in external beam radiotherapy, the emergence of intensity-modulated techniques and new protocols for altered fractionation have pushed renewed interest on the potential use of very high dose-rate in radio-response in certain treatment settings [16, 17]. A detailed insight on the DR effects in *in vivo* experiments with pulsed irradiation (FLASH) has been given by Favaudon et al [24]. However, our source turned out to be radically different with respect to pulse length and energy range (this one more comparable for instance with the IntraBeam^®^) and it gave us momentum to *in vitro* investigate the irradiation effects of a Plasma Focus source. The pulsed plasma device under evaluation, a “Mather type” Plasma Focus (Plasma Focus for Medical Applications #3, PFMA-3) has been recently developed at the University of Bologna (Montecuccolino Laboratory) for a possible application to radiotherapy treatment of malignant cells. PFMA-3 has been geared as a pulsed X-rays generator. The low-energy (up to 200 keV) X-rays produced by conversion on a brass target of the self-collimated electron beam generated by the device during the pinch phase are able to deliver a very high DR as shown in Table 1 where the main PFMA-3 features are summarized [25].

RETRACTED

**Table 1:** Technical characteristics of the PFMA-3 source.

PFMA-3 main working parameters [26, 27]	
Operating Voltage [kV]	18
Primary Electron Bunch [mC]	0.1
Primary Electron Spectrum Energy Bulk [keV]	50–80
Photon Spectrum Energy Bulk [keV]	30–60
Pulse Duration [s]	20×10−9–50×10^−9^
Pulse Frequency [Hz]	0.1*

*Actual working value without cooling system.

PFMA-3 is superior in terms of intensity and DR in comparison with other standard technologies like LINACs and X-rays tubes. PFMA-3 is able to deliver a dose of the order of 0.2–1 Gy/pulse, each pulse lasting 20 to 50 × 10^−9^ sec. On the contrary, other technologies can generally reach fractions of Gy in the order of one second or more (see Table 2).

**Table 2:** Comparison between the PFMA-3 [26, 28] and other technologies. Given the energy range, a direct evaluation against X-ray sources can be made [27, 29]. LINACs [16, 30] sources here added as reference, have higher energies than PFMA-3 and constitute a widespread technology and a common standard for radiotherapy.

	PFMA-3*	X-RAY TUBE	LINAC
ACCELERATED PARTICLES (AP)	Electrons	Electrons	Electrons
E__MAX_AP_ [keV]	300	400	25×10^3^
BEAM	X-Rays	X-Rays	X-Rays
DOSE RATE [GY s^-1^]	10^7^	< 10^−1^	< 1
GY PER PULSE	0.2–1		
COST [€]	3×10^5^	<10^5^	10^6^–10^7^

*PFMA-3 is able to deliver 10^15^ electron per shot. The PF phenomena arising in the so called “pinch phase” [28] are in the range of the tens of nanoseconds.

In the present study, we explored PFMA-3 biological effectiveness on SK-Mel28 and A375, two human melanoma cell lines characterized by radioresistance [31] in comparison with a conventional X-ray tube (XRT), calibrated to mimic the PFMA-3 energy spectrum. Little is known about molecular effects of very high DR. This report is, at our knowledge, the first attempt to describe the advantages of such dose rates on enhancing melanoma cells radiosensitivity through the study of biological effects.

## Materials and methods

### Radiation sources

High-DR (order of 0.2–1 Gy per shot, each shot lasting 20–50 ns) experiments were performed with the PFMA-3 device (Montecuccolino Laboratory, University of Bologna). The Monte Carlo simulation of the X-ray spectrum exhibited a component at 10 keV, and a component at 50 keV with a tail of up to 200 keV [32]. The dose assessment delivered in each shot has been extensively validated using Gafchromic^®^ films (EBT2/3) [26]. It was referred from dose measurements that photons reaching the cell layer had energies above 30 keV. Low-DR (order of 10^-1^Gy min^-1^) experiments were performed with a BALTEAU CSC320/70 X-ray tube (COMECER S.p.A.-ACCREDIA LAT 065), with a mean energy spectrum of 37.3 keV. Taking into account that the X-ray device had an affective dose-rate delivery of approximately 0.2 Gy/min and that the PFMA-3 delivered its dose of nearly 0.2–0.3 Gy/shot in few tens of ns with one minute for cooling between shots, the “total exposure time” for the two devices could be considered comparable.

RETRACTED

### Cell culture

The human skin melanoma cell lines SK-Mel28 and A375 were obtained from the ATCC (Catalog number: HTB-72) and from Istituto Zooproflilattico Sperimentale della Lombardia e dell’Emilia Romagna (Catalog number: BS TCL 88) respectively. They were both cultured as recommended. They were grown on 25–175 cm^2^ tissue culture flasks containing Dulbecco’s modified Eagle’s medium (DMEM), supplemented with 10% heat-inactivated fetal bovine serum, 1% L-glutamine and 0.5% penicillin/streptomycin (all reagents were purchased by Sigma-Aldrich, St Louis, MO, USA). Cells were maintained in a humified 5% CO_2_ air incubator at 37°C. Twenty-four hrs before irradiation cells were harvested at near confluence with 0.1% trypsin (Sigma-Aldrich). Cells were plated at the same density as a monolayer on Mylar^®^ foils positioned in a special holder for irradiation. They were irradiated with 2, 4, 8 Gy under PFMA-3 and comparatively under XRT. Control and irradiated cells were subsequently detached, counted and then seeded according to the experimental timeline schedule (up to 120hrs).

### Annexin V-fluorescein isothiocyanate (FITC)/propidium iodide (PI) staining and cell cycle analysis

To determine the extent of apoptosis induction after radiation treatment, flow cytometric analysis of Annexin V-FITC/PI-stained samples was performed using AnnexinV-FITC Apoptosis detection kit (eBioscience Dx Diagnostics, Vienna, Austria) as previously reported [33]. Cell cycle analysis was carried out using a PI/RNaseA staining according to standard procedures. All the flow cytometric analyses were performed on an FC500 flow cytometer (Beckman, Miami, FL, USA), with the appropriate software (CXP, Beckman).

### Western blot analysis

Western blot analysis were performed as previously detailed [34]. Cells were lysed using the M-PER Mammalian Protein Extraction Reagent, supplemented with the Protease and Phosphatase Inhibitor Cocktail (Thermo Fisher Scientific Inc., Rockford, IL, USA). Equivalent amounts of protein in each sample (about 40 μg) were separated by gradient gels (4%–20% acrylamide). Analysis with an antibody to β-actin documented equal protein loading. Antibodies to caspase-9 (#9508, 1:1000, anti–mouse), caspase -8 (#9927, 1:1000, anti–mouse), Bcl-xL (#2762, 1:1000, anti–rabbit), cyclin B1 (#4138, 1:1000, anti–rabbit), E-Cadherin (#3195, 1:1000, anti–rabbit), Phospho-p53 (Ser15) (#9284, 1:1000, anti–rabbit), β-actin (#8457, 1:1000, anti–rabbit) were all from Cell Signaling Technology (Danvers, MA, USA).

RETRACTED

### Clonogenic assay

Control and treated cells were seeded in 6-well plates at 500–5000 cells per well (four replicates of each sample) with 3 ml complete medium. Cells were incubated to allow colony formation and medium was changed every three days. After 9 days, cells were washed twice with phosphate–buffered saline (PBS), fixed with 10% formaldehyde (Sigma) and stained with 0.01% (w/v) crystal violet (Sigma-Aldrich, Steinheim, Germany). Air–dried colonies containing more than 50 individual cells were counted under a stereomicroscope (Bausch & Lomb, Rochester, NY, USA). The Plating Efficiency (PE) was calculated by dividing the number of counted colonies by the number of seeded cells. The Surviving Fraction (SF) was calculated by normalizing the PE values of irradiated samples to PE values of corresponding control and a survival curve was generated.

### Senescence assay

Ninety-six hrs after irradiation control and treated cells were seeded onto a glass slide. Beta galactosidase activity at pH 6 was detected using a Senescence Cells Histochemical Staining Kit (Sigma-Aldrich, St. Louis, MO). The assay was performed according to the manufacturers´ instructions. Senescent cells were detected by formation of local blue precipitate upon enzymatic cleavage under a Leitz Orthoplan light microscope (LM, Leica Microsystem Inc., Bannockburn, Ill, USA) [35].

### DNA double-strand breaks assay

Three, 24 and 48 hrs after irradiation control and treated cells were seeded on glass slides. Cells were fixed with 4% formaldehyde for 10 min at room temperature and washed three times with PBS. To permeabilize the cells, the slides were submersed in a glass jar over a 10-min period with 0.2% Triton X100 in PBS. The slides were washed three times in PBS. Then, the slides were incubated in blocking solution (5% bovine serum albumin in PBS) for 1 hour at room temperature. Primary anti-pospho-Histone-H2A.X (Ser139) (Merck Millipore KGaA, Darmstadt, Germania) incubation was carried out in 1% bovine serum albumin PBS solution overnight at 4 °C (1:1000). After three washing steps, cells were then incubated in the secondary antibody FITC-conjugated (DAKO Denmark A/S Glostrup, Denmark) for 1 hour at room temperature (dilution 1/30). The slides were washed three times and the nuclei were counterstained with DAPI (final working concentration of 1 μg/ml in Vectashield). The slides were covered with coverslips and stored in the dark at– 20°C. Images were taken under a Zeiss Axio Imager.Z1 microscope (Zeiss, Jena, Germany), with 40x/NA 0.75 optics, coupled to a computer-driven Zeiss AxioCAM digital camera (MRm), using the Zeiss AxioVision (version 4.5) software.

RETRACTED

### Wound healing assay

The *in vitro* scratch wound experiments were performed according to previous studies [36]. Briefly, control and treated cells were seeded in 6-well plates (four replicates of each sample) with 3 ml complete medium and allow reaching confluence. A reproducible longitudinal scratch in the monolayer was made the following day using sterile micropipette tips. The process of wound closure was monitored at different time points (0, 6, 21, 30, 45 hrs) by photographing the central field of the scratches under an inverted light microscopy (Olympus CKX41, Olympus Corp, Tokyo, Japan) mounted with a digital camera (C-7070 Wide Zoom, Olympus) at 10 × magnification. The pictured field was standardized each time against a horizontal line drawn on the base of the plate passing through the center of each well. Morphometric analysis of cell migration was performed by one experienced investigator blinded to the specific experimental conditions using a computerized image analysis system (Qwin, Leica Microsystem Imaging Solution, Ltd). A region of 2.58 x 10^6^μm^2^ that included the artificial scratch and the adjacent cell monolayer was selected as the standard region of interest. The wound healing effect was calculated as (1-A*x*/A0) %, where A0 and A*x* represented the empty scratch area at 0 and *x* hours, respectively.

### Glutathione and lipid peroxidation analyses

For detection of intracellular glutathione, SK-Mel28 were incubated (30 min, 37° C) with 60 μM monochlorobimane (mBCl). This non-enzymatic fluorescent reagent when bound to reduced (GSH) or oxidized (GSSG) glutathione, formed the adduct bimane–glutathione (B-SG), that emitted a fluorescent blue light (Ex/Em = 380nm/461nm), whereas mBCl unbound was almost non-fluorescent. For the detection of lipid peroxidation on cells membrane, SK-Mel28 were incubated (30 min, 37° C) with 1 mM boron-dipyrromethene (BODIPY). Oxidation of the polyunsaturated butadienyl portion of the dye resulted in a shift of the fluorescence emission peak from ~590 nm to ~510 nm. Fluorescence images of 100 × magnification were acquired under the epifluorescence microscope Nikon Eclipse Ti-E (Nikon Instruments Europe B.V., Bologna, Italy). Scanning electrochemical microscopy (SECM) measurements were performed using an experimental setup coupling a 910B SECM (CHI Instruments, USA) with a Nikon Ti optical microscope (Nikon Instruments Europe B.V., Bologna, Italy). All electrochemical measurements were carried out in a 35 mm Petri dish located on the plate holder of the inverted microscope and used to allocate the Mylar^®^. The SECM probes were 10 μm diameter platinum ultra-microelectrodes (UMEs). The RG value of all the Pt UMEs used in the present work was 10. An Ag/AgCl/3 M KCl electrode was used as a reference electrode and a platinum wire as the counter electrode. The translational rate of the UME for the SECM images was 25 μm/s.

RETRACTED

### Statistical analysis

The data were presented as the mean values from at least three separate experiments ± SD or SEM. Statistical analyses were performed using Student’s t test at a significance level of P <0.05 (GraphPad Prism Software).

## Results

### 1) PFMA-3 very high dose rate caused radiation-induced clonogenic cell death greater than XRT

SK-Mel28 and A375 cells were irradiated at a high DR (pulses of 0.2 Gy in 20 to 50 ×10^−9^ sec) by PFMA-3 and, in the same experimental conditions, by the XRT device calibrated to mimic PFMA-3 energy spectrum. Cells were seeded 20 hrs before irradiation and treated at 2, 4 and 8 Gy. We examined the anti-proliferative effect of the two X-ray sources through clonogenic assay, the “gold standard” for radiation effect studies. Fig 1a showed the dose-response curves for cell killing induction. In response to PFMA-3 irradiation, the survival fractions at 2 Gy (SF2) were 0.19 for SK-Mel28 and 0.40 for A375; in contrast XRT SF2 were nearly 1 for SK-Mel28 and 0.66 for A375. PFMA-3 SF4 and SF8 decreased to 0.04 and 0.02 for SK-Mel28 and to 0.07 and 0.06 for A375 respectively.

**Fig 1:** PFMA-3 causes radiation-induced clonogenic cell death greater than XRT. **(a)** Colony forming unit assay on SK-Mel28 and A375 cells irradiated with PFMA-3 and XRT at 2, 4 and 8 Gy. Data are representative of three independent experiments performed in triplicate and SD is not shown being less than 10%. Black (SK-Mel28) and red (A375) asterisks indicate statistically significant differences (*P<0.05, **P <0.005). **(b)** Radiobiological parameters of SK-Mel28 and A375 cell lines for PFMA-3 and XRT 2, 4, 8 Gy irradiation. SF2, SF4 and SF8 survival fraction at 2, 4 and 8 Gy respectively. D50, 50% survival dose. The D50 values for XRT device were used as standard reference for the RBE evaluations. The MLQ curve has been built from parameters suggested for SK-Mel28 and for low energy X-ray sources with a correction for the exposure time [37].

RETRACTED

Instead, for the XRT device the SF4 and SF8 were 0.53 and 0.12 for the SK-Mel28 and 0.28 and 0.22 for the A375. The survival curves for SK-Mel28 were fitted using a modified standard linear quadratic model [20] to evaluate 50% survival dose(D50). D50 values for SK-Mel28 were 1.25 Gy for PFMA-3 and 4.3 Gy for XRT, confirming that PFMA-3 treatments were more effective than XRT ones to decrease ability of SK-Mel28 to form a clone (Fig 1b). D50 values for A375 were 1.6 Gy for PFMA-3 and 2.7 Gy for XRT. In Fig 1b we also reported the relative biological effect, RBE, evaluated relative to 50% survival using, as standard reference, the XRT radiation.

### 2) PFMA-3 very high dose rate induced a more severe DNA damage with respect to XRT

Induction of DNA double-strand breaks (DNA-DSB) is one of the key mechanisms underlying IR antiproliferative effect. A very early step in the cellular response to DSB is the phosphorylation at serine 139 of a histone H2A variant, H2A.X, at the sites of DNA damage [4]. Pospho-H2A.X at Ser139 was detected by immunofluorescence and analyzed under microscope. SK-Mel28 samples treated with 2 Gy PFMA-3 showed a great pospho-H2A.X fluorescence after 3 hrs. This DNA damage tended to disappear at 24 and 48 hrs. Interestingly, 2 Gy XRT treatment induced a lower damage at 3 hrs (Fig 2a). Also in A375 samples 2Gy PFMA-3 irradiation caused a higher H2A.X phosphorylation in comparison to XRT (Fig 3a).

**Fig 2:** PFMA-3 causes a DNA-DSB more severe with respect to XRT in SK-Mel28. Induction of DSB was assessed through detection of phosphorylation of H2A.X at Ser139 (green) by immunofluorescence and microscopy analysis. **a)** DSB after 2 Gy treatment. **b)** DSB after 4 Gy treatment. **c)** DSB after 8 Gy treatment. ctrl, control cells. **d)** Western blot analysis documenting phospho-p53 (Ser51) levels modulation in PFMA-3 and XRT irradiated samples. Antibody to b-actin served as a loading control. ctrl, control cells.

**Fig 3:** PFMA-3 causes a DNA-DSB more severe with respect to XRT in A375. Induction of DSB was assessed through detection of phosphorylation of H2A.X at Ser139 (green) by immunofluorescence and microscopy analysis. a) DSB after 2 Gy treatment. b) DSB after 4 Gy treatment. c) DSB after 8 Gy treatment. ctrl, control cells. d) Western blot analysis documenting phospho-p53 (Ser51) levels modulation in PFMA-3 and XRT irradiated samples. Antibody to b-actin served as a loading control. ctrl, control cells.

Four and 8 Gy PFMA-3 caused a similar damage with respect to 2 Gy treatment at 3 hrs in SK-Mel28 cells but the effect lasted longer, until 24 and 48 hrs. In 4 and 8 Gy XRT samples we observed a significantly less pronounced increase of phospho-Ser139 H2A.X at all time points (Fig 2b and 2c). At 4 and 8 Gy also A375 trend was similar to SK-Mel28 (Fig 3b and 3c). It is well known that tumor suppressor protein p53 is a central stress protein in DNA damage response [38]. We studied the effects of PFMA-3 and XRT irradiation on the phosphorylation status of p53 at Ser15 in our cell models. In SK-Mel28 western blot analysis documented that PFMA-3 was able to enhance Ser15 p-p53 at all doses. On the contrary, XRT did not induce a p-p53 increase but rather a little inhibition respect to control (Fig 2d). Also for A375 cells it was evident that PFMA-3 enhanced Ser15 p-p53 levels, mostly at 8 Gy. XRT treatment confirmed its weak effect (Fig 3d). Taken together these results clearly showed that PFMA-3 induced a greater, less easy-to-repair DNA-DSB and a consequent more important p53 activation in comparison to XRT in both cell lines.

RETRACTED

### 3) PFMA-3 and XRT treatments did not induce significant apoptotic events until 96 hours

IR therapy, like other types of anticancer treatments, may induce multiple forms of cell death. Apoptosis is the major modality observed in response to irradiation. It is mostly induced in hematopoietic cells or in p53 wildtype tumor cells, but it is well known that final cell death mode is determined by the type of radiation, the dose of radiation and the molecular profile of the cells [39, 40]. Through flow cytometry analysis we evaluated whether the antiproliferative effects observed could be related to apoptosis. Fig 4a showed analysis of Annexin V-FITC/PI-stained SK-Mel28 irradiated with 2 Gy PFMA-3 and XRT.

**Fig 4:** PFMA-3 and XRT treatments did not induce significant apoptotic events until 96 hours. Flow cytometric analysis of Annexin V-FITC/PI-stained SK-Mel28 cells treated with **a)** 2 Gy **b)** 4 Gy **c)** 8 Gy PFMA-3 and XRT at different time points. The percentages of early apoptotic cells (Annexin V FITC+/PI-), late apoptotic/necrotic cells (Annexin V FITC+/PI+) and necrotic cells (Annexin V FITC-/PI+) were plotted. The histograms were representative of three separate experiments. Asterisks indicated statistically significant differences (**P <0.005). ctrl, control cells. **d)** Western blot analysis documenting some apoptotic marker levels modulation in PFMA-3 and XRT irradiated samples. Antibody to b-actin served as a loading control. ctrl, control cells.

Cells were followed for 96 hrs from irradiation and no significant enhancement in the percentage of early apoptotic (single positive for Annexin V) and/or late apoptotic (double positive for Annexin V and PI) cells was detected, neither with PFMA-3, nor with XRT. In addition, 4 Gy irradiation did not induce important increase of Annexin V positive cells (Fig 4b). Analysis of 8 Gy treated samples showed a higher percentage of necrotic cells (PI positive), both in PFMA-3 and XRT but only at 96 hrs the difference was statistically significant (Fig 4c). Western blot analysis of some apoptotic markers, caspase-9, -8 and Bcl-XL in PFMA-3 and XRT 2, 4 and 8 Gy treated cells correlated with flow cytometric studies. These data suggested that up to96 hrs of treatment apoptosis was not the SK-Mel28 primary process of death after irradiation (Fig 4d).

RETRACTED

### 4) PFMA-3 very high dose rate altered SK-Mel28 cell cycle distribution more severely than XRT and finally induced the appearance of a sub-G1 peak

To better characterize biological effects of the very high DR delivered on cancer cells survival, we proceeded to consider irradiation cytostatic effects through cell cycle distribution analysis. In 2 Gy PFMA-3 treated cells cytostatic effects were weak, because a moderate accumulation in the G2/M phase (about 24%) was visible only after 96 hrs. Two Gy XRT cells did not show any significant effect in cell cycle distribution (Fig 5a).

**Fig 5:** PFMA-3 very high dose rate altered SK-Mel28 cell cycle distribution more severely than XRT and finally induced the appearance of sub-G1 peak. Flow cytometric analysis of cell cycle distribution in SK-Mel28 cell line treated with **a)** 2 Gy **b)** 4 Gy **c)** 8 Gy PFMA-3 and XRT for different times. The histograms were representative of three separate experiments. ctrl, control cells. **d)** Western blot analysis documenting cyclin-B1 levels modulation in PFMA-3 and XRT irradiated cells. Antibody to b-actin served as a loading control. ctrl, control cells.

Conversely, in 4 Gy PFMA-3 samples a real cell cycle arrest in the G2/M phase (about 50%) occurred already after 24 hrs and lasted until 120 hrs. Very interestingly, the 4 Gy XRT treatment was not able to produce this effect (Fig 5b). Eight Gy treated sample analysis showed a greater G2/M arrest, about 60% after 24 hrs and, at 120 hrs, sub-G1 peak (apoptotic cells) reached about 24% (Fig 5c). Even at this high dose, XRT cytostatic effect was weak and much lower in comparison with PFMA-3. Therefore, at early times and up to 96 hrs, in SK-Mel28 the prevailing PFMA-3 effect consisted in cellular cell cycle shift to G2/M phase, preceding by a few hours the display of the peculiar endonucleases-induced DNA cuts, liable for the appearance of sub-G1 peak. These results have been molecularly strengthened through western blot analysis of the levels of cyclin B1 that, together with cdc2, forms the mitosis-promoting factor (MPF). Fig 5d showed that PFMA-3 irradiation induced a cyclin B1 decrease at all doses and mostly at 24 hrs after treatment. It was well known that cyclin B1 reduction correlates with G2/M arrest [40]. In contrast, after XRT treatment (at all doses) cyclin B1 levels remained constant. These results elucidated that PFMA-3 antiproliferative prevalence was due to cytostatic instead of cytotoxic effects.

RETRACTED

### 5) PFMA-3 very high dose rate caused higher levels of stress-induced premature senescence with respect to XRT

Having noted the consistent G2/M arrest concurrently with the absence of evident apoptotic effects, we hypothesized that a stress-induced premature senescence (SIPS) might account for the greater effect of PFMA-3. In fact, it has been demonstrated that as well as an irreversible arrest in the G1 phase of the cell cycle [41, 42], senescence could also be induced during a prolonged G2 arrest [43–45]. Therefore, senescence activated β-gal (SA- β-gal) activity was measured (at 96 hrs) through a histochemical staining kit, X-gal based. Two, 4 and 8 Gy PFMA-3 samples expressed a number of β-gal positive cells significantly higher than control cells and respect to XRT samples (Fig 6).

**Fig 6:** PFMA-3 caused higher levels of SIPS respect to XRT. Representative images of staining for senescence-associated β-galactosidase 96 hrs following irradiation with 2, 4 and 8 Gy PFMA-3 and XRT. Data were representative of three independent experiments. ctrl, control cells.

### 6) PFMA-3 very high dose rate affected cell migration properties more than XRT

We performed scratch wound-healing assay to evaluate very high DR effects also on SK-Mel28 and A375 migration ability. This assay is a commonly accepted and well-developed method to measure cell migration *in vitro* [46, 47]. After irradiation cells were seeded and, once the proper confluence reached, they were scratched. The process of wound closure, driven by the migration of cells into the wounded area, was monitored under stereomicroscope at different time points until 45 hrs after scratching. Figs 7a and 8 showed that repair in XRT samples was always greater than in PFMA-3 at all doses and all time points for both cell lines.

**Fig 7:** PFMA-3 affected SK-Mel28 migration abilities more than XRT. **a)** Cell migration behaviour was evaluated during performance of a wound-healing assay after treatment with 2 Gy, 4 Gy and 8 Gy PFMA-3 and XRT. Data were representative of three independent experiments performed in quadruplicate. ctrl, control cells. Asterisks indicated statistically significant differences (*P <0.05, **P <0.005, ***P <0.0005). **b)** Western blot analysis documenting E-cadherin levels modulation in PFMA-3 and XRT irradiated samples. b-actin loading control was not shown. ctrl, control cells.

RETRACTED

**Fig 8:** PFMA-3 affected A375 migration abilities more than XRT. Cell migration behaviour was evaluated during performance of a wound-healing assay after treatment with 2 Gy, 4 Gy and 8 Gy PFMA-3 and XRT. Data were representative of three independent experiments performed in quadruplicate. ctrl, control cells. Asterisks indicated statistically significant differences (*P <0.05, **P <0.005, ***P <0.0005).

In particular, for SK-Mel28 XRT maximum repair (60%) was obtained at 2 Gy after 45 hrs (at the same time control sample repair was 73%), whereas PFMA-3 maximum repair was about 40%. A375 trend was very similar. We completed this analysis with an expression study of E-cadherin protein levels after irradiation in SK-Mel28 samples. Epithelial cadherin (E-cadherin) is a major cell-cell adhesion molecule that interconnects epithelial cells [48–50]. In cancer cells, the loss or decrease in E-cadherin expression and/or function typically correlates with high invasiveness and metastasis [49, 50]. After 2 Gy PFMA-3 treatment, E-cadherin levels increased (at 24 hrs). This enhancement was more evident in 4 Gy PFMA-3 samples (24 hrs) and raised again in 8 Gy PFMA-3 ones. On the contrary, levels of E-cadherin were reduced with respect to control, after all doses XRT irradiation (Fig 7b). Taken together these data suggested that very high DR played a role also in SK-Mel28 and A375 migration/invasiveness mechanisms.

### 7) PFMA-3 very high dose rate increased glutathione and lipid peroxidation more than XRT

It is well known that IR can directly interact with target macromolecules or indirectly with water, leading to a radiolysis process and to the generation of reactive oxygen and nitrogen species (ROS/RNS) that can affect several cellular functions, such as the mitochondrial metabolism [51]. The transient cellular response to the induced oxidative stress (protective mechanism) is strongly correlated to the radiation dose and quality [51]. The reducing agent glutathione (GSH) is considered a free radical scavenger while it is converted into its oxidized form glutathione disulfide (GSSG) [52]. The synthesis and metabolism of GSH are well balanced within the cell and their alteration can compromise the defense against ROS [53]. In order to evaluate how the DR of the impacting radiation is critical in determining an effect on the oxidative and metabolic balance we investigated the variation of glutathione levels and the lipid peroxidation in irradiated cells compared to control. Fig 9a showed that the fluorescence of the adduct bimane–glutathione (B-SG) induced in SK-Mel28 after PFMA-3 irradiation was higher, in a dose dependent manner, than after XRT treatment.

RETRACTED

**Fig 9:** PFMA-3 induced glutathione and lipid peroxidation production greater than XRT. **a)** Visualization of the SK-Mel28 living cells 3 hrs after irradiation with PFMA-3 or XRT (at 2 and 4 Gy) and of those non irradiated (ctrl) loaded by the fluorescent dyes monochloromobimane (mBCl) and boron-dipyrromethene (BODIPY) for a qualitative GSH and lipid peroxidation detection, respectively. Epifluorescence images at 100 × of magnification. **b)** Representative FcMeOH/SECM images in constant height mode of non irradiated (ctrl) and irradiated SK-Mel28 cells at 4 Gy by PFMA-3 and XRT. The regeneration currents recorded were reported as a percentage increase/decrease of the signal in respect to the one recorded at the same tip-dish distance but far away from cells (I_T_/I_Tdish_). **c)** Histogram reported the values obtained by computing the mean (± SEM) regeneration current recorded on 4 different cells selected from the scanning electrochemical microscopy images. Asterisks indicated statistically significant differences (*P <0.05).

Since monochlorobimane (mBCl) only qualitatively indicates the glutathione levels between compared samples, we also performed scanning electrochemical microscopy (SECM) experiments capable to specifically quantify the GSH levels of each sample. In Fig 9b and 9c the images and the graphs of regeneration currents at SECM ultramicroelectrode measured employing ferrocene-methanol (FcMeOH) redox mediator for control (ctrl), PFMA-3 and XRT irradiated cells were reported. The regeneration currents are strictly correlated to GSH/GSSG levels. In particular, increase of the regeneration current is associated to increased levels of GSH/GSSG ratio and coupled with the capacity of specific enzymes (glutathione dehydrogenase and glutathione reductase) to regenerate the redox mediator GSH. The higher positivity of the mBCl test and the larger regeneration currents found 3 hrs after PFMA-3 irradiation suggested a radiation-induced increment of the GSH levels. We also detected by the boron-dipyrromethene (BODIPY) fluorescent adduct (Fig 9a) a raise of the lipid peroxidation. The GSH/GSSG ratio and the lipid peroxidation of the XRT irradiated cells did not appear to differ significantly from that of the control cells indicating that the radiation effect is DR dependent.

## Discussion

Improvements in RT over the last decade are linked to the emergence of intensity-modulated techniques (IMRT) that modify DR treatment delivery and to the use of proton or heavy ions species [54]. Hadrontherapy and proton radiotherapy have recently attracted growing interest. In fact, superior ballistic properties of charged particles with respect to photons can be translated in higher dose conformity and less involvement of healthy tissue. However, the need for cost reduction is driving the development of new, more compact and economic technologies. The PFMA-3 device was designed to produce a thin plasma leaf through the fast and synchronized discharge of the capacitor bank. When the plasma leaf collapses in the so-called “pinch”, the plasma reaches thermonuclear conditions of pressure and energy density for a few tenths of nanoseconds (Table 1). Depending on the chamber filling gas, nitrogen in our experiments, several kinds of radiation fields are produced. Among those, a naturally collimated electron beam is driven to collide with a target to produce X-Rays. This electron bunch is very intense (0.1 mC) with 10^15^ electrons produced [13]. It is this fast and impressive production that makes the difference, in terms of DR, with other technologies. Moreover, PFMA-3 manufacturing, utilization and radiation protection arrangements require quite low costs in contrast to the high application flexibility (Table 2). Preliminary data about antitumor efficacy of PFMA-3 have been obtained in glioblastoma (T98G cell line) [12] and breast cancer preclinical models (MCF-7 cell line) [13]. Although the effects of an important DR variation after low-LET radiation has been reported for several years [55], up to now limited recent biological data have been published on very high DR effect in tumor. The present work hypothesized that the very high DR delivered by PFMA-3 significantly impaired radioresistant melanoma survival in comparison with a conventional XRT. As indicated by CFU assay, PFMA-3 treatment had a higher antiproliferative power with respect to XRT. In particular, the D50 (50% survival dose) was 3.4 fold and 1.7 fold lower than the XRT D50 for SK-Mel28 and A375 respectively. These values are very interesting and it would be worthwhile to deeply investigate them in comparison with the heavier charged particles. This could have important therapeutic implications because tumor could be treated with lower total doses, hence with likely lower incidence of radiation-induced damage to healthy tissues. We described how PFMA-3 antiproliferative effect resulted by a greater and less easy-to-repair DNA-DSB and a consequent higher p53 activation in both cell lines. As showed by Annexin V flow cytometric analysis and by caspases and Bcl-XL western blot assessment, apoptotic cell death was not the principal inhibitory effect exerted by both sources on SK-Mel28 line, at least until 96 hrs. The preferential response to IR seemed to be the cell cycle arrest and the premature senescence induction [56–58], Cell cycle distribution and SA- β-gal activity studies elucidated that, in SK-Mel28, PFMA-3 prevalence emerged in connection with cytostatic rather than cytotoxic effects. The immunofluorescence and electrochemical analyses revealed that higher levels of GSH and a greater lipid peroxidation were induced by the PFMA-3 source, corroborating the view that SIPS is aneffect of the oxidative stress and that cellular senescence is a mechanism of radiosensitization likely induced by a ROS-mediated DNA damage [59] DR dependent. Finally, our characterization showed that PFMA-3 impaired both cell lines migration properties more than XRT and this was confirmed by the parallel increase of E-cadherin levels (in SK-Mel28). Since it is well known that the adhesion of cells to extracellular matrix (ECM) as well as to other cells can positively modulate the resistance to RT [60, 61] our results implicated that a lower migration capability could also express a lower radioresistance. The present study confirmed the innovative features of DR and therefore of the radiation source for the optimization of radiotherapy application. However further experiments and a more specific approach are required to establish mechanistic molecular basis of the observed PFMA-3 superior biological effects.

RETRACTED

## Conclusions

With this *in vitro* characterization, we provided a contribution to understanding the greater effectiveness of ultra-high dose rate energy delivery in impairing proliferation of melanoma cell lines SK-Mel28 and A375, known to be resistant to radiation damage. These preliminary results represent an encouraging first step for future preclinical characterizations. This work could also have important future perspectives for the development of a novel class of Plasma Focus technology-based devices, therapeutically performing, with low costs and established technologies.
